# Prediction of Renal Function Damage in Patients with Essential Hypertension Based on Stepwise Regression Equation Scanning by AASI

This article has been retracted.

**DOI:** 10.1155/2022/4728921

**Published:** 2022-05-28

**Authors:** Yaqiong Wu, Guangyu Ma, Hongzhen Sun, Sijie Zhang, Xingtao Li

**Affiliations:** ^1^The Department of Cardiology, Fourth Hospital of Hebei Medical University, Shijiangzhuang, Hebei 050011, China; ^2^The Department of Haematology, Fourth Hospital of Hebei Medical University, Shijiangzhuang, Hebei 050011, China

## Abstract

Detection of arterial stiffness is an important method to predict the occurrence of hypertension complications and to screen patients with high cardiovascular risk. In order to predict the damage of AASI to the renal function of patients with essential hypertension, the prediction of AASI based on stepwise Regression equation scanning for renal function damage in patients with essential hypertension is proposed. Measure the 24 h ambulatory blood pressure of the selected subjects, establish a linear Regression equation scanning, and calculate the slope of the straight line, and finally, the slope is AASI. According to the quartiles, AASI is divided into four parts: group I < 0.53 (*n* = 49); 0.53 ≤ group II < 0.60 (*n* = 51); 0.60 ≤ group III < 0.69 (*n* = 48); group IV ≥ 0.69 (*n* = 44). Experiment result shows the following: with the increase of AASI, cystatin (CysC) also increased significantly, while CysC-eGFR decreased significantly (*P* < 0.05). Compared with groups I, II, and III, Scr and CysC in group IV increased (*P* < 0.05), and Ccr, CysC-eGFR, and (CKD-EPI)-eGFR all decreased (*P* < 0.05). AASI is positively correlated with CysC performance, and the correlation coefficient *r* is 0.637. It is negatively correlated with Ccr performance, and *r* is -0.361. It is negatively correlated with CysC-eGFR, and *r* is -0.698. And it is negatively correlated with (CKD-EPI)-eGFR, and *r* is -0.331. Age and 24 h PP also showed an increasing trend with the increase of AASI, and it suggests that age may be an influencing factor that promotes kidney damage caused by hypertension; it also suggests that AASI can be used as a new indicator of arterial compliance; AASI is linearly related to various indicators of renal damage and can be used as a predictive indicator of renal damage caused by essential hypertension; cystatin C and the estimated glomerular filtration rate CysC-eGFR based on cystatin C are better than other indicators reflecting glomerular filtration rate, more sensitively assess the degree of early renal damage. Obesity may also be a factor that promotes kidney damage caused by hypertension.

## 1. Introduction

Ambulatory blood pressure monitoring (ABPM) can reflect blood pressure levels and circadian rhythms; there is a good correlation with the damage degree of target organs such as heart, brain, and kidney. It also has important significance in studying the pathogenesis of hypertension-related complications [1]. The ambulatory blood pressure-related arteriosclerosis index is a series of indicators derived from ABPM that reflect the elastic function of arteries; the application scope of AB-PM in clinical has been further expanded [2]. Symmetrical Ambulatory Arterial Stiffness Index (S-AASI) is a new index derived from ABPM to assess arterial stiffness. In the current research, there are not many reports on the correlation between S-AASI and target organ damage in hypertension [3]. AASI is a new indicator of arteriosclerosis discovered by using a series of systolic and diastolic blood pressure values obtained by ABPM to perform function fitting [4]. In response to this research question, Kotecha et al. reported that AASI is positively correlated with PP, and it is less dependent on blood pressure value and blood pressure variability than PP; it is a good supplement to PP predicting arterial elastic function, and it is recommended that AASI.PP and blood pressure variability should be used in combination in the evaluation of arteriosclerosis [5]. Couderc et al. pointed out that AASI is affected by factors such as the correlation between systolic and diastolic blood pressure, age, gender, PP, and nocturnal blood pressure when it reflects the degree of arteriosclerosis and predicts target organ damage; the measurement results are unstable [6]. Turner et al. believe that S-AASI is a newer and improved dynamic arteriosclerosis index; the calculation of S-AASI value is due to the introduction of the concept of symmetric linear Regression equation scanning and the use of *r* value for correction; it is believed to be able to detect arteriosclerosis more accurately; it may be better than AASI in evaluating the correlation with hypertension target organ damage; S-AASI has not been shown to be superior to AASI [7]. Therefore, the pros and cons of the abovementioned indicators for evaluating arteriosclerosis in clinical use are still controversial [8]. On the basis of the current research, the AASI based on the stepwise Regression equation scanning is proposed to predict the renal function damage of patients with essential hypertension. Measure the 24 h ambulatory blood pressure of the selected subjects, establish a linear Regression equation scanning, and calculate the slope of the straight line; finally, the slope is AASI. According to the quartiles, AASI is divided into four parts: group I < 0.53 (*n* = 49); 0.53 ≤ group II < 0.60 (*n* = 51); 0.60 ≤ III group < 0.69 (*n* = 48); IV group ≥ 0.69 (*n* = 44). Age and 24 h PP also showed an increasing trend with the increase of AASI; it suggests that age may be an influencing factor that promotes kidney damage caused by hypertension; it also suggests that AASI can be used as a new indicator of arterial compliance; AASI is linearly related to various indicators of renal damage; it can be used as a predictor of renal damage caused by essential hypertension; cystatin C and the estimated glomerular filtration rate CysC-eGFR based on cystatin C are better than other indicators reflecting glomerular filtration rate, more sensitively assess the degree of early renal damage. Obesity may also be a factor that promotes kidney damage caused by hypertension.

## 2. Method

### 2.1. Research Objects

A total of 192 patients with essential hypertension were selected for the outpatient department of the cardiology department of a university hospital; among them, there are 98 males and 94 females; the age fluctuates in the range of 40-81; the diagnoses of all selected subjects met the selection criteria of this experiment but did not meet the exclusion criteria.

1. *Selection Criteria*. Diagnosed as a patient with essential hypertension, routine urine examination showed negative urine protein, those who did not take antihypertensive drugs within two weeks before seeing a doctor, and understand this experiment and give informed consent
2. *Exclusion Criteria*. People with secondary hypertension, past liver and kidney dysfunction, urinary system diseases, pheochromocytoma, congenital heart disease, valvular disease, severe heart failure, myocardial infarction, atrial fibrillation, pleural or abdominal effusion, severe edema or malnutrition, diabetes, ketoacidosis, hyperthyroidism and hypothyroidism, gout, cerebrovascular accidents, and severe blood system diseases; those who take drugs that affect blood pressure measurement within 2 weeks; and those who have recently undergone glucocorticoid or hemodialysis treatment [9]

### 2.2. Experimental Method

#### 2.2.1. Record Blood Pressure and Calculate AASI

All subjects wore 24 h ambulatory blood pressure monitors, using MOBI-0-GRAPH ambulatory blood pressure monitor. Set the blood pressure to be measured every half an hour from 6 : 00 in the morning, until 23 : 00 at night. Set again from 23 : 00 at night; blood pressure was measured every hour until 6 : 00 a.m. the next day. During the measurement, the patient is required not to stay up late to be consistent with daily life. Establish a linear Regression equation scanning and calculate the slope of the straight line, and finally, the slope is AASI. According to the quartiles, AASI is divided into four parts: group I < 0.53 (*n* = 49); 0.53 ≤ group II < 0.60 (*n* = 51); 0.60 ≤ III group < 0.69 (*n* = 48); IV group ≥ 0.69 (*n* = 44).

#### 2.2.2. Calculate 24 h Pulse Pressure Based on Blood Pressure

Pulse pressure, also known as pulse pressure (PP), is the difference between systolic blood pressure (SBP) and diastolic blood pressure (DBP); it is a commonly used index to evaluate arterial compliance in clinical practice.

#### 2.2.3. General Data Collection

Record the general condition of the patient, such as age, weight, height, and heart rate. And calculate its body mass index (BMI) based on weight and height and the patient's blood glucose, blood lipids, liver function, kidney function, blood routine, urine routine, electrolytes, and other biochemical indicators.

#### 2.2.4. Indicators of Kidney Function

All subjects get blood from fasting veins in the morning, the particle-enhanced transmission immunoturbidimetric method was used to determine the serum cystatin C level of subjects, and bring the measured serum CysC into the corresponding formula for estimating glomerular filtration rate, MacIsaac modified formula: GFR = (77.30/CysC) + 2.32, and calculate CysC-eGFR.

### 2.3. Statistical Processing

The data of this study was processed using the SPSS17.0 statistical software package, statistical analysis adopts a two-sided test, and *P* < 0.05 means the difference is statistically significant, unless otherwise specified. The measurement data is statistically described in the form of mean ± standard deviation ($\bar{x}\pm s$). Counting data is expressed in frequency and percentage. The chi-square test was used for the statistical inference of the comparison between the count data groups, and the analysis of variance was used for the statistical inference of the comparison between the measurement data groups. Pearson correlation analysis was used to compare the linear correlation between AASI and renal damage indexes. In addition, the multiple linear stepwise regression analysis method was used to take the kidney damage index as the dependent variable, and construct a model with base data as independent variables.

## 3. Results and Analysis

### 3.1. Baseline Data Analysis

According to the ambulatory blood pressure value measured at 24 h, take systolic blood pressure and diastolic blood pressure as the abscissa and ordinate, respectively, draw a scatter plot, establish a linear Regression equation scanning, calculate the slope of the straight line, and finally get the AASI with 1-the slope, and according to the quartiles, AASI is divided into four parts: group I: 49 cases, AASI < 0.53; group II: 51 cases, 0.53 ≤ AASI < 0.60; group III: 48 cases, 0.60 ≤ AASI < 0.69; and group IV: 44 cases, AASI ≥ 0.69. After analysis of variance for each group: heart rate between 4 groups, there was no statistically significant difference in BMI comparison (*P* > 0.05), the age difference between the groups was statistically significant (*P* < 0.05), and it is suggested that as the AASI level increases, age is also increasing. The difference in 24 h PP between the groups was statistically significant (*P* < 0.05), suggesting that with the increase of AASI level, 24 h PP also gradually increased.

### 3.2. Single Factor Analysis

Among the indicators of kidney damage, the four groups of data were first analyzed by variance analysis between groups, and the results showed that the differences between the index groups were statistically significant (*P* < 0.05). Then, use the Bonferroni test method to compare the two within the group; the results are as follows: in Scr indicators, there were statistically significant differences between group II and group I, group III and group I, and group IV, group II, and group III (*P* < 0.05). In the CysC index, group II is compared with the group I, and group III is compared with group I and group II; there was a statistically significant difference between group IV and group I, group II, and group III (*P* < 0.05). In the Ccr index, group II is compared with group I, and group III is compared with group I; there was a statistically significant difference between group IV and group I, group II, and group III (*P* < 0.05). In the CysC-eGFR index, group II is compared with group I, and group III is compared with group I and group II; there was a statistically significant difference between group IV and group I, group II, and group III (*P* < 0.05). In the (CKD-EPI)-eGFR index, group II is compared with group I, and group III is compared with group I; there was a statistically significant difference between group IV and group I, group II, and group III (*P* < 0.05). The tip is as follows: as AASI increases, cystatin (CysC) also increased significantly, while CysC-eGFR decreased significantly (*P* < 0.05). Compared with groups I, II, and III, both Scr and CysC in group IV increased (*P* < 0.05), and Ccr, CysC-eGFR, and (CKD-EPI)-eGFR all decreased (*P* < 0.05).

### 3.3. The Linear Correlation between Various Indexes of Renal Function and AASI

The indicators of kidney damage are as follows: creatinine clearance, cystatin C, CysC-eGFR, and (CKD-EPI)-eGFR, respectively, and AASI after linear correlation analysis by Pearson correlation analysis method, AASI is positively correlated with CysC, the correlation coefficient *r* is 0.637; it is negatively correlated with Ccr performance, and *r* is -0.361; it is negatively correlated with CysC-eGFR performance, and *r* is -0.698. It is negatively correlated with (CKD-EPI)-eGFR, and *r* is -0.331. After adjusting for age factors, after partial correlation analysis, AASI is positively correlated with CysC performance and negatively correlated with the performance of Ccr, CysC-eGFR, and (CKD-EPI)-eGFR, the correlation coefficients are as follows, and the *P* values are all <0.05, as shown in Figure 1.

### 3.4. Multiple Linear Regression Analysis of Each Index and AASI

1. Taking CysC as the dependent variable, then use age, heart rate, BMI, and AASI as independent variables, and the multiple linear stepwise regression analysis is shown in Table 1. The result shows the following: the Regression equation scanning of cystatin C and AASI is as follows: CysC = 0.657 + 2.111 × AASI.

(2) Taking Ccr as the dependent variable, then use age, heart rate, BMI, and AASI as independent variables; the multiple linear stepwise regression analysis is shown in Table 2. The Regression equation scanning of creatinine clearance rate and AASI, age, and BMI is as follows: Ccr = 120.012 − 39.885 × AASI − 0.898 × age − 1.211 × BMI.

(3) Taking CysC-eGFR as the dependent variable, then use age, heart rate, BMI, and AASI as independent variables; the multiple linear stepwise regression analysis is shown in Table 3; the result shows the following: the Regression equation scanning of CysC-eGFR and AASI is as follows: CysC − eGFR = 121.598 − 157.968 × AASI.

(4) Taking (CKD-EPI)-eGFR as the dependent variable, then use age, heart rate, BMI, and AASI as independent variables; the multiple linear stepwise regression analysis is shown in Table 4; the result shows the following: the Regression equation scanning of (CKD-EPI)-eGFR, AASI, and age is as follows: (CKD‐EPI) − eGFR = 130.011 − 35.010 × AASI − 0.603 × age.

The kidneys can regulate blood pressure; it can also be damaged by persistent high blood pressure. There is an interaction between high blood pressure and the kidneys; actively control benign hypertension (especially moderate to severe benign hypertension); it is very important to prevent kidney damage caused by hypertension. How does the kidney perform the task of regulating blood pressure? First of all, the kidneys regulate the balance of water and electrolytes in the body; if the kidneys are damaged, water and sodium cannot be excreted from the body; it will cause increased blood vessel pressure and blood pressure. Secondly, the endocrine function of the kidney, the renin, and angiotensin that it secretes are involved in regulation, human blood pressure, and once the kidney is damaged, the imbalance of these endocrine hormones can cause vascular tension and cause high blood pressure. Kidney damage caused by long-term high blood pressure, it is also due to the continuous state of high blood pressure, which continuously damages the blood vessel wall, gradually lead to arteriosclerosis, and after arteriosclerosis, changes in hemodynamics, less blood flowing into the kidneys, eventually cause kidney damage [10].

This study found that the dynamic arteriosclerosis index (AASI) is linearly related to various indicators of renal damage [11]. As a new indicator of arteriosclerosis, AASI predicts changes in vascular disease earlier and more sensitively than pulse pressure; it mainly reflects the degree of arteriosclerosis. As mentioned earlier, the higher the degree of arteriosclerosis, the closer the AASI is to 1. The better the arterial elasticity, the closer the AASI is to 0 [12]. The pulse pressure mainly depends on the ejection rate of the left ventricle, the stroke volume of the heart, and factors such as the compliance of the large arteries and the pressure reflection waves of the peripheral blood vessels, and as the pulse pressure increases, its damage to blood vessels is also strengthened; the tube wall is in a state of high tension for a long time; it is easy to fatigue and break, and the factor that regulates the vasoconstriction and relaxation function is out of proportion, and vascular endothelial dysfunction strengthens the progression of vascular sclerosis; therefore, pulse pressure has a certain role in reflecting the degree of arteriosclerosis [13]. As obtained from this experiment, according to the AASI grouping, as the AASI level increases, 24 h PP is gradually increasing, but the stability of PP is weaker than that of AASI and is susceptible to changes in blood pressure fluctuations and other factors and affects the accuracy of prediction, so the AASI in this study has become the most suitable indicator for predicting arteriosclerosis [14].

According to the results of this experimental study, AASI can be used as a predictor of renal damage in patients with essential hypertension; at present, a large amount of data has proved that AASI can predict the damage of target organs; for example, it can predict cardiovascular and cerebrovascular diseases, especially the predictive value of stroke is greater. The ambulatory arteriosclerosis index (AASI) is calculated from ambulatory blood pressure monitoring, and ABPM is since the 1960s, one of the important results of studying hypertension; it is required that in daily life, according to the set time interval, it can automatically measure blood pressure, and the series of blood pressure values obtained include daytime activity and night sleep; it objectively reflects the dynamic changes of human blood pressure [15]. Hypertensive target organ damage (TOD) is a possible result in the development of hypertension; therefore, actively predict the target organ damage caused by hypertension, and intervene in a timely manner; it is of great significance to delay the occurrence of target organ damage [16]. According to research findings, AASI has been confirmed as a predictor of renal damage caused by essential hypertension. AASI is greatly affected by age, the systolic and diastolic blood pressure of normal people slowly increase with age, mainly because the peripheral resistance of blood vessels also increases with age, and for the elderly, the increase in systolic blood pressure is mainly caused by the gradual hardening of the aorta with age and the gradual decrease in the vascular volume of the elastic large arteries; its diastolic blood pressure is reduced, mainly because the amount of blood injected into the periphery from the heart during systole increases, at the beginning of diastole, as the amount of blood remaining in the aorta decreases, and the elasticity of the arteries is weakened, and diastolic blood pressure decreases [17]. And get older with age, human aging, the thickness of the media in the aorta increases, and the elastic fibers become thinner, increasing the stiffness of the aorta; therefore, the results of this study are significantly due to the focus on the predictive value of the dynamic arteriosclerosis index on the renal damage caused by essential hypertension; to summarize the results of this research, AASI is positively correlated with CysC performance and negatively correlated with Ccr, CysC-eGFR, and (CKD-EPI)-eGFR performance. It shows that with the influence of long-term hypertension, the AASI gradually increases, that is, the compliance of the arteries gradually decreases, and the degree of hardening gradually increases, and kidney damage is also gradually getting worse. After adjusting for age factors, after partial correlation analysis, AASI is positively correlated with CysC performance and negatively correlated with Ccr, CysC-eGFR, and (CKD-EPI)-eGFR performance; the *P* values are all <0.05, indicating the error that may be caused by excluding the age factor, and AASI and renal damage indicators are correlated [18]. Further analyze the multiple linear stepwise regression model, and the result shows that for every 0.01 increase in AASI, cystatin C increased by 0.02 mg/L, creatinine clearance decreased by 0.40 mL/(min · 1.73m^2^), CysC-eGFR decreased by 1.58 mL/(min · 1.73m^2^), and (CKD-EPI)-eGFR decreased by 0.35 mL/(min · 1.73m^2^) (all *P* values < 0.05), and controlling the confounding factors of age and body mass index, it further illustrates that AASI can be used as an independent predictor of renal damage in patients with essential hypertension. But in this multiple linear stepwise regression analysis, we also found that the creatinine clearance rate decreases by 0.90 mL/(min · 1.73m^2^) for every 1 year increase in age, (CKD-EPI)-eGFR decreased by 0.60 mL/(min · 1.73m^2^) (all *P* values < 0.05), and this also suggests that age may also be a factor that promotes kidney damage caused by primary hypertension. In addition, we also found that for every increase in body mass index (BMI) by 1 unit, creatinine clearance decreased by 1.21 mL/(min · 1.73m^2^); this also shows that obesity may also be a factor that promotes kidney damage caused by primary hypertension. And Table 4 of the results of this study also shows that AASI has the strongest correlation with cystatin C and CysC-eGFR (*r* = 0.637; *r* = −0.698); tip in the experiment is only in the indicators of cystatin C and CysC-eGFR that the differences in each group were statistically significant.

## 4. Conclusion

Propose the prediction of renal damage in patients with essential hypertension based on AASI stepwise Regression equation scanning, select qualified subjects to measure 24 h ambulatory blood pressure to calculate AASI, AASI is linearly related to various indicators of renal damage, and it can be used as a predictor of renal damage caused by essential hypertension. Age and 24 h PP also showed an increasing trend with the increase of AASI, it suggests that age may be an influencing factor that promotes kidney damage caused by hypertension, and it also suggests that AASI can be used as a new indicator of arterial compliance. Obesity may also be a factor that promotes kidney damage caused by hypertension. Cystatin C and the estimated glomerular filtration rate CysC-eGFR based on cystatin C are more sensitive to assess the degree of early renal damage than other indicators reflecting glomerular filtration rate.

## Figures and Tables

**Figure 1:** The linear correlation between various indexes of renal function and AASI.

**Table 1:** Results of multiple linear regression with CysC as the dependent variable.

*X*	*B* value	Standard error	Beta	*P*
Constant	0.657	0.080	-	*P* < 0.001
AASI	2.111	0.145	0.633	*P* < 0.001

**Table 2:** Results of multiple linear stepwise regression with Ccr as the dependent variable.

*X*	*B* value	Standard error	Beta	*P*
Constant	120.012	10.120	-	*P* < 0.001
AASI	-39.012	7.111	-0.259	*P* < 0.001
Age	-0.898	0.079	-0.551	*P* < 0.01
BMI	-1.211	0.229	-0.320	*P* < 0.05

**Table 3:** Results of multiple linear stepwise regression with CysC-eGFR as the dependent variable.

*X*	*B* value	Standard error	Beta	*P*
Constant	121.598	4.149	-	*P* < 0.001
AASI	157.968	9.910	-0.721	*P* < 0.001

**Table 4:** Results of multiple linear stepwise regression with (CKD-EPI)-eGFR as the dependent variable.

*X*	*B* value	Standard error	Beta	*P*
Constant	130.011	7.972	-	*P* < 0.001
AASI	-35.010	6.729	-0.282	*P* < 0.001
Age	-0.603	0.072	-0.420	*P* < 0.01

## Data Availability

The data used to support the findings of this study are available from the corresponding author upon request.
